This article has been retracted.

# A Case-Cohort Study of Cadmium Body Burden and Gestational Diabetes Mellitus in American Women

**DOI:** 10.1289/ehp.1408282

**Published:** 2015-02-24

**Authors:** Megan E. Romano, Daniel A. Enquobahrie, Christopher D. Simpson, Harvey Checkoway, Michelle A. Williams

**Affiliations:** 1 Department of Epidemiology, Brown University, Providence, Rhode Island, USA; 2 Department of Epidemiology, University of Washington, Seattle, Washington, USA; 3 Center for Perinatal Studies, Swedish Medical Center, Seattle, Washington, USA; 4 Department of Environmental and Occupational Health Sciences, University of Washington, Seattle, Washington, USA; 5 Department of Family and Preventive Medicine, University of California, San Diego, La Jolla, California, USA; 6 Department of Epidemiology, Harvard T.H. Chan School of Public Health, Boston, Massachusetts, USA

## Abstract

**Background:**

Environmental cadmium (Cd) exposure is associated with type 2 diabetes. However, the association of Cd and gestational diabetes mellitus (GDM) is unknown.

**Objectives:**

We examined the association between body burden of Cd and GDM risk.

**Methods:**

We used 140 GDM cases and 481 randomly selected noncase subcohort members from the Omega Study to conduct a case-cohort study. Creatinine (Cr)–corrected Cd in early pregnancy urine (U-Cd) was measured by inductively coupled plasma mass spectrometry. Tertiles (< 0.29; 0.29–0.42; ≥ 0.43 μg/g Cr) were defined using the subcohort’s U-Cd distribution. GDM was diagnosed using the 2004 American Diabetes Association guidelines. Adjusted odds ratios (ORs) and 95% confidence intervals (CIs) were estimated using logistic regression.

**Results:**

GDM cases had higher geometric mean U-Cd (0.39 μg/g Cr; 95% CI: 0.37, 0.41) than noncases (0.31 μg/g Cr; 95% CI: 0.29, 0.33). Odds ratios for GDM increased with increasing U-Cd tertile (OR = 1.64; 95% CI: 0.88, 3.05 for middle vs. low tertile; OR = 2.07; 95% CI: 1.15, 3.73 for high vs. low tertile; *p*-trend = 0.015). Overweight/obesity (body mass index ≥ 25 kg/m^2^) did not modify the association between U-Cd and GDM (*p* = 0.26).

**Conclusions:**

Our findings suggest that body burden of Cd increases risk of GDM in a dose-dependent manner. Improved understanding of environmental factors influencing GDM may facilitate early identification of women at high risk of GDM.

**Citation:**

Romano ME, Enquobahrie DA, Simpson CD, Checkoway H, Williams MA. 2015. A case-cohort study of cadmium body burden and gestational diabetes mellitus in American women. Environ Health Perspect 123:993–998; http://dx.doi.org/10.1289/ehp.1408282

## Introduction

Gestational diabetes mellitus (GDM), a pregnancy-related glucose intolerance disorder, complicates up to 14% of pregnancies each year in the United States [American Diabetes Association (ADA) 2004]. GDM increases the lifetime risk of type 2 diabetes mellitus, obesity, and metabolic syndrome for both the mother and her infant (ADA 2004; Metzger 2007). Although some strong risk factors for GDM are known [e.g., maternal age (Cypryk et al. 2008) and high prepregnancy body mass index (BMI) (Torloni et al. 2009)], less is understood about environmental risk factors.

Cadmium (Cd) is widely used in commercial products, including batteries, pigments, and plastics. Mining, industrial processing, burning of coal, and household wastes all contribute to occupational exposure and the entry of Cd into the environment [Agency for Toxic Substances and Disease Registry (ATSDR) 2012]. Cd has a high rate of soil-to-plant transfer, and the general population is exposed to Cd primarily via ingestion of food and inhalation of tobacco smoke (ATSDR 2012; Järup and Åkesson 2009). Although relatively low levels of Cd are found in most foods, there is relatively high Cd content in grains, shellfish, and organ meats. (Järup and Åkesson 2009). Additionally, regular ingestion of eggs, cereals, leafy greens, and yams have been associated with greater Cd body burden among premenopausal women (Adams et al. 2011). Cd is readily stored in the leaves of tobacco plants, and cigarette smokers are exposed to high levels of Cd via inhalation (ATSDR 2012). Cd exposure has been associated with renal damage (Kido et al. 2003), cardiovascular disease (Tellez-Plaza et al. 2013), osteoporosis (Engström et al. 2012), and cancer (Julin et al. 2012).

Although Cd accumulates primarily in the kidney and liver, pancreatic tissue also accumulates Cd to a lesser degree, and elevations in pancreatic Cd have been correlated with reductions in serum insulin among rats exposed to Cd (Edwards and Prozialeck 2009). Diabetogenic effects of Cd have been demonstrated in experimental studies (Edwards and Prozialeck 2009; Lei et al. 2007). Rodent models suggest that Cd may impair insulin secretion via damage to pancreatic β-cells in the islets of Langerhans (Chang et al. 2013; Chen et al. 2009; El Muayed et al. 2012).

A growing body of evidence from population-based studies suggests an association between body burden of Cd and type 2 diabetes. Several (Afridi et al. 2008, 2013; Haswell-Elkins et al. 2007; Kolachi et al. 2011; Schwartz et al. 2003), but not all (Barregard et al. 2013; Moon 2013; Swaddiwudhipong et al. 2010, 2012), studies among nonoccupationally Cd-exposed study participants have suggested an association between higher levels of Cd and type 2 diabetes. In addition to clinically recognized diabetes, higher body burden of Cd has also been associated with impaired fasting glucose in a dose-dependent fashion (Schwartz et al. 2003). To the best of our knowledge, the relation between body burden of Cd and GDM risk has not been investigated previously. The objective of this case-cohort study was to examine whether elevated body burden of Cd is associated with an increased risk of GDM. We assessed arsenic as a potential confounder because arsenic has been associated with increased risk of GDM (Ettinger et al. 2009) and was an important co-exposure in our study setting (King County Environmental Health Services 2010). We also explored whether observed associations with Cd were modified by prepregnancy BMI because overweight or obese women are known to have increased risk of GDM (Torloni et al. 2009).

## Methods

*Study population and setting*. The Omega Study, a large (*n* = 4,344) prospective cohort study (1996–2008) based at the Center for Perinatal Studies at Swedish Medical Center in Seattle, Washington, was designed to investigate risk factors for pregnancy complications (Qiu et al. 2011). Participants were recruited from prenatal care clinics affiliated with Swedish Medical Center (Seattle) and Tacoma General Hospital (Tacoma, Washington). Women who spoke English and initiated prenatal care at a study clinic before 20 weeks gestation were eligible for participation. Women who were < 18 years of age, did not intend to carry the pregnancy to term, or did not plan to deliver at study institutions were excluded. All procedures and study protocols were approved by the institutional review boards at the University of Washington and the study hospitals, and all participants provided written informed consent.

We conducted a case-cohort study nested in the Omega Study cohort. We selected a reference subcohort of 750 women randomly drawn from the full cohort. The initial case group included all 190 diagnosed GDM cases from the full cohort. Among the randomly selected members of the subcohort, 44 were GDM cases. Women were excluded for the following reasons: Urine samples were not available for 18 subcohort members, 17 women in the subcohort had preexisting diabetes mellitus, 1 subcohort member had missing GDM case status, 6 subcohort members and 4 GDM cases had renal disease, 27 noncases and 10 GDM cases had multiple fetal births, 9 subcohort members delivered before 24 weeks gestation, and 8 women had Cd values suggestive of renal impairment (> 2 μg/g Cr) (Kido et al. 2003). Finally, we excluded one subcohort member with urinary creatinine > 300 mg/dL and 138 subcohort members and 36 GDM cases with urinary creatinine < 30 mg/dL (Figure 1), per World Health Organization (WHO) guidelines, which suggest that creatinine concentration may be used to identify spot urine samples that are too concentrated (> 300 mg/dL) or too dilute (< 30 mg/dL) to provide valid estimates of the concentration of the urinary chemical of interest [International Programme on Chemical Safety and World Health Organization (IPCS and WHO) 1996]. The characteristics of women with dilute urine did not differ substantially from those included in the analytic population, except that fewer GDM cases with low creatinine had normal prepregnancy BMI (18.5 to < 25 kg/m^2^) (44.4% vs. 50.7%; *p* = 0.02) and more were underweight before pregnancy (BMI < 18.5 kg/m^2^) versus GDM cases with creatinine 30–300 mg/dL (5.6% vs. 1.4%; *p* = 0.05). This is in line with previous reports that low creatinine is common among individuals with reduced lean body mass (Barr et al. 2005). After exclusions, the analytic population included 621 women (481 noncase subcohort members and 140 GDM cases).

**Figure 1:** Exclusions based on missing exposure or gestational diabetes mellitus (GDM) information, medical history, and pregnancy characteristics.

*Data collection*. Information on sociodemographic characteristics, reproductive and medical histories, lifestyle factors (such as alcohol and tobacco use), and maternal anthropometry was collected by trained interviewers using a structured questionnaire shortly after enrollment (15 gestational weeks, on average). Participants completed a self-administered, validated, and semiquantitative food-frequency questionnaire (FFQ) describing nutritional intake over the prior 6 months (3 months before pregnancy through the first 3 months of pregnancy, on average) (Patterson et al. 1999). Maternal medical records were abstracted by trained study personnel to confirm medical and reproductive histories and to ascertain pregnancy course, complications, and outcomes.

*Cadmium and arsenic exposure assessment*. At 15 weeks gestation, on average (SD = 2.9; interquartile range = 13–17 gestational weeks), a clean-catch spot urine sample was collected in polyethylene containers, promptly separated into 2-mL aliquots, and stored at –80°C until analysis. Urine heavy metal concentrations, including Cd and total arsenic, were quantified using a validated method of inductively coupled plasma–mass spectrometry (ICP-MS) following published protocols (Heitland and Koster 2004) at Metametrix Clinical Laboratory, a Clinical Laboratory Improvement Amendments (CLIA)–certified facility in Duluth, Georgia. Briefly, urine samples were shaken and 1 mL was acidified with 1% HNO_3_ (100 μL). An internal standard solution containing scandium, rhodium, and germanium (500 μL) was added. Samples were diluted to 5 mL with deionized water. Polyatomic interferences were minimized by using ICP-MS with a dynamic reaction cell (PerkinElmer SCIEX Elan DRC II with ESI SC-4, FAST Autosampler). The accuracy of ICP-MS was checked by conducting proficiency testing using urine reference material (New York Toxic/Trace Elements in Urine Event #1 2012). Urinary creatinine (Cr) concentration was assessed using a commercially available kit (Genzyme Diagnostics, Catalogue #221-30/#221-50) with improved Jaffe reaction. The limits of detection for urinary Cd and total arsenic were 0.12 and 3.0 μg/g Cr, respectively. Total arsenic in urine reflects both organic and inorganic species of arsenic. Speciated arsenic would have been preferable since organic arsenic species are in general less toxic than inorganic forms and recent ingestion of seafood increases the level of organic arsenic in urine (Orloff et al. 2009). Therefore, we adjusted for self-reported fish consumption in all models that included total urinary arsenic. Laboratory personnel were blinded to GDM case status.

*GDM diagnosis*. As part of routine antenatal follow-up of all women at participating clinics, a 50-g, 1-hr oral glucose challenge test was administered between gestational weeks 24 and 28 to screen for GDM. Women who failed the screening test [glucose ≥ 7.8 mmol/L (≥ 140 mg/dL)] completed a diagnostic 100-g, 3-hr oral glucose tolerance test within 2 weeks of the screening test. Women were diagnosed with GDM if two or more 100-g, 3-hr oral glucose tolerance test levels exceeded ADA 2004 criteria: fasting ≥ 5.3 mmol/L (≥ 95 mg/dL); 1-hr ≥ 10.0 mmol/L (≥ 180 mg/dL); 2-hr ≥ 8.6 mmol/L (≥ 155 mg/dL); 3-hr ≥ 7.8 mmol/L (≥ 140 mg/dL) (ADA 2004).

*Statistical analysis*. We compared the frequency distribution of relevant characteristics of the population between GDM cases and the subcohort. Tertiles were defined based upon the distribution of urinary creatinine–corrected Cd (U-Cd) in the subcohort. Unconditional logistic regression was used to assess the risk of GDM across tertiles of U-Cd. The case-cohort odds ratio (OR), calculated using the logit-link function, is a good estimate of the incidence proportion ratio in cumulative-incidence type case-cohort studies that include thorough case ascertainment from the full population (Kass and Gold 2005; Prentice 1986), such as the present study. Additionally, logistic regression has been successfully used for prior case-cohort studies that did not use time-to-event data (Chevrier et al. 2011). We conducted trend tests using the median value within each tertile of U-Cd as the score variable. Covariates were entered into each model one at a time, and we compared adjusted and unadjusted ORs to assess confounding. We retained covariates in the final models that substantially altered unadjusted ORs (> 10% change) and the following variables selected based on *a priori* knowledge of their associations with exposure (Cd body burden) and outcome (GDM): maternal age (years), prepregnancy BMI (kilograms per meter squared), nulliparity (yes/no), family history of diabetes (yes/no), and maternal race (non-Hispanic white, yes/no). GDM in a prior pregnancy (yes/no), current preeclampsia (yes/no), chronic hypertension (yes/no), family history of hypertension (yes/no), marital status (married, yes/no), post high school education (yes/no), smoking during pregnancy (yes/no), urinary total arsenic (U-As), and iron-deficiency anemia during pregnancy (yes/no) were evaluated as potential confounding variables. All models that contained arsenic included further adjustment for average servings of fish per week based upon FFQ. Adjusted ORs and 95% confidence intervals (CIs) were calculated from the models.

*Secondary analyses*. We evaluated potential effect modification by prepregnancy BMI by examining the independent and joint effects of high U-Cd (≥ 0.29 μg/g Cr, representing the combined middle and high tertiles of U-Cd) and prepregnancy overweight/obese status (BMI ≥ 25 kg/m^2^) on GDM risk and adding a term for the interaction between high U-Cd and prepregnancy overweight/obese status to the multivariable model. GDM risk among women with high U-Cd was compared with GDM risk among women with low U-Cd (< 0.29 μg/g Cr) within groups defined by prepregnancy overweight/obese status (prepregnancy BMI 18.5 to < 25 kg/m^2^ vs. ≥ 25 kg/m^2^). We also examined whether the joint effect of U-Cd and prepregnancy overweight/obesity status on risk of GDM was greater than expected, given their independent effects. For these analyses, we categorized women as *a*) low U-Cd and normal prepregnancy BMI (reference), *b*) high U-Cd and normal prepregnancy BMI, *c*) low U-Cd and overweight/obese prepregnancy BMI, and *d*) high U-Cd and overweight/obese prepregnancy BMI. Women who were underweight (prepregnancy BMI < 18.5 kg/m^2^) were excluded from this analysis (31 subcohort members, 2 GDM cases).

Because smoking tobacco cigarettes is a major potential source of Cd exposure in the general population (ATSDR 2012), and GDM risk is increased among smokers (England et al. 2004), we performed a sensitivity analysis including ever versus never smoking and an interaction term for U-Cd and smoking status in the multivariable model. Sensitivity analyses were also conducted including participants with samples that were deemed dilute (< 30 mg/dL) according to the WHO guidelines (619 noncase subcohort members; 176 GDM cases) (IPCS and WHO 1996), because the WHO guidelines are potentially overly restrictive for female populations (Barr et al. 2005). Because micronutrient deficiencies, including calcium, zinc, and iron, increase Cd absorption (Kippler et al. 2009), we conducted an exploratory analysis to assess whether dietary intake of essential micronutrients [total daily dietary calcium, iron (total iron, heme iron, or nonheme iron), and zinc intake] or for falling below the Institute of Medicine’s recommended dietary allowance for pregnant women (< 1,000 mg/day calcium, < 27 mg/day iron, < 11 mg/day zinc) (Institute of Medicine Panel on Micronutrients 2001) influenced the association between Cd and GDM. Finally, we conducted an exploratory analysis assessing the risk of GDM across tertiles of U-As, defined according to the distribution in the subcohort. The multivariable logistic regression model included adjustment for age, prepregnancy BMI, race/ethnicity, nulliparity, preeclampsia, chronic hypertension, family history of diabetes, family history of hypertension, U-Cd, and fish consumption.

All statistical analyses used robust standard error estimates, used the alpha level of 0.05 to define statistical significance, and were completed using STATA version 12.0 (StataCorp, College Station, TX, USA).

## Results

Women with GDM were older (33.6 vs. 32.8 years), had greater prepregnancy BMI (27.0 vs. 23.7 kg/m^2^), and reported sedentary behavior more often (9% vs. 4%) than women without GDM (Table 1). Compared to women without GDM, fewer GDM cases were non-Hispanic white (69% vs. 84%). Women with GDM had a higher frequency of preeclampsia (8% vs. 2%), chronic hypertension (9% vs. 4%), and a positive family history of diabetes (34% vs. 15%) or hypertension (63% vs. 45%) compared with women without GDM. There were no significant differences between women with and without GDM in terms of parity, educational attainment, marital status, smoking habits, average weekly servings of fish, gestational week at urine collection, or total urinary arsenic concentrations (Table 1).

**Table 1:** Characteristics of the study population according to gestational diabetes status.

Covariate	Noncases in subcohort	Gestational diabetes cases	*p*-Value
*n*	481	140
Maternal age (years)	32.8 ± 4.5	33.6 ± 4.7	0.05
Prepregnancy BMI (kg/m^2^)	23.7 ± 5.0	27.0 ± 7.2	0.05
Underweight (< 18.5)	30 (6)	2 (1)
Normal weight (18.5 to < 25.0)	312 (65)	71 (51)
Overweight (25.0 to < 30.0)	100 (21)	36 (26)
Obese (≥ 30.0)	38 (8)	31 (22)
Parity
Nulliparous	282 (59)	77 (55)
Parous	199 (41)	63 (45)
Race/ethnicity			0.05
Non-Hispanic white	402 (84)	97 (69)
Other race/ethnicity	79 (16)	42 (30)
Education
Post–high school education	434 (90)	131 (94)
High school or less	17 (4)	8 (6)
Marital status
Married	408 (85)	116 (83)
Unmarried	73 (15)	24 (17)
Preeclampsia^*a*^			0.05
Yes	12 (2)	11 (8)
No	467 (97)	127 (91)
Iron-deficiency anemia^*a*^
Yes	9 (2)	6 (4)
No	467 (97)	134 (96)
Chronic hypertension			0.05
Yes	18 (4)	13 (9)
No	463 (96)	127 (91)
Family history of diabetes^*b*^			0.05
Yes	70 (15)	47 (34)
No	411 (85)	93 (66)
Family history of hypertension^*c*^			0.05
Yes	216 (45)	88 (63)
No	265 (55)	52 (37)
Smoking status^*d*^
Never	316 (66)	94 (67)
Ever	134 (28)	37 (26)
Leisure time physical activity			0.05
Yes	432 (90)	119 (85)
No	18 (4)	12 (9)
Average weekly servings of fish (*n*)^*e*^	1.3 ± 1.2	1.3 ± 1.2
Gestational week of spot urine collection	15.2 ± 2.9	15.0 ± 2.9
Urinary measurements [GM (95% CI)]
Cadmium (μg/g Cr)	0.31 (0.29, 0.33)	0.39 (0.37, 0.41)
Total arsenic (μg/g Cr)	22.8 (21.2, 24.5)	25.5 (22.0, 29.5)
Creatinine (mg/dL)	83.6 (79.5, 87.9)	82.6 (75.3, 90.7)
Abbreviations: Cr, creatinine; GM, geometric mean. Values are mean ± SD or *n* (%). ^***a***^During study pregnancy. ^***b***^Any primary or secondary family member with type 1 or type 2 diabetes. ^***c***^Any primary or secondary family member with chronic hypertension. ^***d***^Self-reported smoking status. ^***e***^Dietary intake estimated from semiquantitative food frequency questionnaire.			

The geometric mean of Cd (0.31 μg/g Cr; 95% CI: 0.29, 0.33) was slightly lower among women without GDM vs. women with GDM (0.39 μg/g Cr; 95% CI: 0.37, 0.41) (Table 1). Women in the middle tertile (0.29–0.42 μg/g Cr) for U-Cd had an elevated, but not statistically significant risk of GDM (OR = 1.64; 95% CI: 0.88, 3.05), compared with those in the lowest tertile (< 0.29 μg/g Cr) (Table 2). Women in the highest tertile for U-Cd (≥ 0.43 μg/g Cr) had two times the risk of GDM, compared with those in the lowest tertile (OR = 2.07; 95% CI: 1.15, 3.73). We observed a statistically significant trend of increasing risk of GDM with greater U-Cd (*p*-trend = 0.015) (Table 2).

**Table 2:** Odds ratios for the association between tertiles of urinary cadmium and risk of gestational diabetes.

Urinary cadmium (μg/g creatinine)^*a*^	*n*	*n* (%)^*b*^	OR^*c*^ (95% CI)
Low (< 0.29)	197	32 (16.2)	1.00 (reference)
Middle (0.29–0.42)	200	44 (22.0)	1.64 (0.88, 3.05)
High (≥ 0.43)	212	52 (24.5)	2.07 (1.15, 3.73)
*p*-Trend			0.015
^***a***^Cutoffs for tertiles are based upon the distribution of urinary cadmium among members of the subcohort. ^***b***^*n* (%) with gestational diabetes within tertile of exposure. ^***c***^Adjusted for age, pre-pregnancy body mass index (kg/m^2^), race/ethnicity, nulliparity, preeclampsia, chronic hypertension, family history of diabetes, family history of hypertension, total urinary arsenic, and fish consumption.			

*Secondary analyses*. Among women with normal prepregnancy BMI, 18.5 to < 25 kg/m^2^, women with high U-Cd (≥ 0.29 μg/g Cr) had 2.15 times the risk of GDM compared with women with low U-Cd (< 0.29 μg/g Cr) (OR = 2.15; 95% CI: 1.02, 4.53), whereas among overweight/obese women (prepregnancy BMI ≥ 25 kg/m^2^) women with high U-Cd had 1.21 times the risk (OR = 1.21; 95% CI: 0.58, 2.52) (Table 3). Compared with women who had low U-Cd and normal prepregnancy BMI, women who had high U-Cd and were overweight/obese before pregnancy had 3.5 times the risk of GDM (OR = 3.46; 95% CI: 1.54, 7.78). However, the interaction was not statistically significant (*p*-value = 0.259) (Table 3).

**Table 3:** Interaction of overweight/obesity status and urinary cadmium on risk of gestational diabetes.

Urinary cadmium (μg/g creatinine) [BMI (kg/m^2^)]^*a*^	*n*	*n* (%)^*b*^	OR^*c*^ (95% CI)	OR^*c*^ (95% CI)
Low (< 0.29) [18.5 < BMI < 25]	102	10 (9.8)	1.00 (reference)	1.00 (reference)
High (≥ 0.29) [18.5 < BMI < 25]	236	49 (20.8)	2.15 (1.02, 4.53)	2.15 (1.02, 4.53)
Low (< 0.29) [BMI ≥ 25]	69	17 (24.6)	1.00 (reference)	2.86 (1.17, 7.61)
High (≥ 0.29) [BMI ≥ 25]	103	33 (32.0)	1.21 (0.58, 2.52)	3.46 (1.54, 7.78)
*p* for ϒ^*d*^				0.259
^***a***^Using the cutoffs for tertiles based upon the distribution of urinary cadmium in the subcohort, women were characterized as have low urinary cadmium (< 0.29 μg/g Cr) or high urinary cadmium (≥ 0.29 μg/g Cr, representing the combined middle and high tertiles). ^***b***^*n* (%) with gestational diabetes within urinary cadmium and prepregnancy BMI group. ^***c***^Model includes adjustment for age, race/ethnicity, nulliparity, preeclampsia, chronic hypertension, family history of diabetes, family history of hypertension, total urinary arsenic, and fish consumption and a term for the interaction between overweight/obese status and cadmium body burden. See “Secondary analyses” for details on the different linear combinations. ^***d***^ϒ = interaction between overweight/obese status and cadmium body burden.				

In the sensitivity analysis assessing smoking status, the interaction between Cd and smoking status was not statistically significant (*p* = 0.56). The odds ratios for GDM risk among never smokers were OR = 1.31 (95% CI: 0.65, 2.64) for middle versus low tertile, and OR = 1.83 (95% CI: 0.94, 3.60) for high versus low tertile; and among ever smokers were OR = 3.09 (95% CI: 0.74, 12.82) for middle versus low tertile, and OR = 3.30 (95% CI: 0.84, 12.89) for high versus low tertile, controlling for age, prepregnancy BMI, race/ethnicity, nulliparity, preeclampsia, chronic hypertension, family history of diabetes, family history of hypertension, U-As, and fish consumption. In secondary analyses related to micronutrient deficiencies, point estimates similar to the main analysis were observed when we excluded the 15 women with iron-deficiency anemia (OR = 1.61; 95% CI: 0.84, 3.07 for the middle vs. low tertile; OR = 2.18; 95% CI: 1.18, 4.02 for the high vs. low tertile; *p*-trend = 0.01) or added adjustment for iron deficiency anemia to the final multivariable model (OR = 1.67; 95% CI: 0.89, 3.11 for the middle vs. low tertile; OR = 2.09; 95% CI: 0.89, 3.11 for the high vs. low tertile; *p*-trend = 0.01). Control for any combination of total daily dietary calcium, iron (total iron, heme, or nonheme), and zinc intake, or for falling below the Institute of Medicine’s recommended dietary allowance for pregnant women (< 1,000 mg/day calcium, < 27 mg/day iron, < 11 mg/day zinc) (Institute of Medicine Panel on Micronutrients 2001) also had no substantial impact on the observed estimates (data not shown).

For the sensitivity analysis that included women with dilute urine (Cr < 30 mg/dL), increases in GDM risk were attenuated and became statistically nonsignificant [OR = 1.19; 95% CI: 0.72, 1.97 for middle (0.21–0.42 μg/g Cr) vs. low (0.21–0.42 μg/g Cr) tertile; OR = 1.34; 95% CI: 0.83, 2.19 for high (0.21–0.42 μg/g Cr) vs. low tertile; *p*-trend = 0.223]. No trend in GDM risk was observed across tertiles of U-As [OR = 0.61; 95% CI: 0.32, 1.13 for middle (16–28 μg/g Cr) vs. low (< 16 μg/g Cr) tertile; OR = 1.15; 95% CI: 0.67, 1.95 for high (≥ 29 μg/g Cr) vs. low tertile; *p*-trend = 0.577].

## Discussion

In our study population, the body burden of Cd was associated with increased risk of GDM in a dose-dependent manner, after accounting for other known risk factors, including arsenic exposure. Women with high U-Cd had twice the risk of GDM as women with low U-Cd. Although the interaction between Cd and overweight/obese status was not statistically significant, the association of higher U-Cd with increased GDM risk was stronger among women who were not overweight/obese before pregnancy.

To our knowledge, no prior epidemiologic research has specifically addressed the association between Cd and GDM. However, a few (Afridi et al. 2008, 2013; Haswell-Elkins et al. 2007; Kolachi et al. 2011; Schwartz et al. 2003), but not all (Barregard et al. 2013; Moon 2013; Swaddiwudhipong et al. 2010, 2012), epidemiologic studies suggest that Cd is associated with type 2 diabetes. Almost all previous research in this area has been cross-sectional (Afridi et al. 2008; Haswell-Elkins et al. 2007; Kolachi et al. 2011; Schwartz et al. 2003; Swaddiwudhipong et al. 2010) or retrospective (Afridi et al. 2013), except for one study that included limited prospective follow-up after cross-sectional assessment (Barregard et al. 2013) and a longitudinal study using change in prevalent diabetes from baseline to 5-year follow-up as an outcome measure (Swaddiwudhipong et al. 2012). Despite this lack of prospective studies, prior research consistently supports the potential for an association between increasing Cd and risk of type 2 diabetes. Research conducted among diverse populations suggests that both men and women with type 2 diabetes have statistically significantly higher levels of Cd in blood (Afridi et al. 2008; Kolachi et al. 2011), urine (Afridi et al. 2008; Haswell-Elkins et al. 2007; Kolachi et al. 2011; Schwartz et al. 2003), and hair (Afridi et al. 2013; Kolachi et al. 2011) compared with those without type 2 diabetes. The most compelling evidence comes from a cross-sectional study conducted by Schwartz et al. (2003) who used data from NHANES III (Third National Health and Nutrition Examination Survey, 1988–1994) to assess whether increased U-Cd was associated with impaired fasting glucose [plasma fasting glucose 6.1 mmol/L (110 to < 126 mg/dL)] and type 2 diabetes among men and women in the United States. A dose-dependent increase in risk was observed across tertiles of U-Cd (0–0.99, 1.00–1.99, ≥ 2 μg Cd/g Cr) for both impaired fasting glucose (OR = 1.48; 95% CI: 1.21, 1.82 for middle vs. low tertile; OR = 2.05; 95% CI: 1.42, 2.95 for high vs. low tertile; *p*-trend < 0.0001) and type 2 diabetes (OR = 1.24; 95% CI: 1.06, 1.45 for middle vs. low tertile; OR = 1.45; 95% CI: 1.07, 1.97 for high vs. low tertile; *p*-trend < 0.0001) (Schwartz et al. 2003).

Although we did not observe evidence of effect modification of the Cd-GDM relation by BMI, we did observe a slightly stronger Cd-GDM association among women who had normal BMI before pregnancy than among women who were overweight/obese before pregnancy. To the best of our knowledge, no other study has examined effect modification of the Cd-diabetes association by BMI. Future studies are needed to clarify the influence of prepregnancy BMI on the Cd-GDM relation.

Development of either GDM or type 2 diabetes represents the interaction of environmental exposures, lifestyle factors, and genetic predisposition. The pathogenesis of both conditions can be thought of as a continuum of dysglycemia with the development of impaired insulin secretion and insulin resistance as a common pathogenic link. The mechanism of Cd-induced diabetes remains uncertain, but appears to involve damage to the insulin-producing β-cells in the islets of Langerhans; such cells in the pancreas of Cd-exposed rats secrete substantially less insulin than those of rats that were not exposed to Cd (Chen et al. 2009). Likewise in cultured rat pancreatic β-cells, Cd increased reactive oxygen species, inducing oxidative stress, and catalyzing cell death (Chang et al. 2013). Alternatively, diabetes-related changes in renal function or other pathophysiologic aspects of impaired glucose tolerance may increase either urinary excretion of Cd or increase body burden of Cd in humans. Although reverse causation is unlikely because we measured U-Cd early in pregnancy, before most GDM-related changes to metabolism or renal function, it cannot be completely ruled out.

One prior study suggests that chronic exposure to arsenic is also a risk factor for GDM (Ettinger et al. 2009). Ettinger et al. (2009) observed that women with high total arsenic blood levels (2.09–24.07 μg/L) had almost three times the odds (OR = 2.8; 95% CI: 1.1, 6.9) of impaired glucose tolerance [blood glucose > 7.8 mmol/L (> 140 mg/dL)] compared with women with the lowest arsenic levels (0.23–0.92 μg/L). In an exploratory analysis of our data, there was no apparent trend between increasing tertiles of U-As and GDM risk after adjustment for other potential risk factors. There may, however, be residual confounding by arsenic exposure in our Cd-GDM analysis, because our measure of total arsenic in urine may not adequately reflect the toxicologically relevant arsenic species. Further, spot urine samples may not capture the totality of arsenic exposure across pregnancy, because variability in U-As excretion and metabolite distribution occurs over the course of pregnancy (Hopenhayn et al. 2003), whereas U-Cd levels are stable throughout pregnancy (Hernandez et al. 1996).

Although Cd absorption increases among women with calcium, zinc, and/or iron deficiencies (Kippler et al. 2009), adjustment for iron deficiency anemia or low dietary intake of micronutrients did not substantially alter the association observed between U-Cd and GDM in this population. More sensitive metrics of calcium, iron, and zinc status, such as blood measures (Shvetsov et al. 2009), may be necessary to elucidate the complex interrelationship among essential and toxic metals and GDM risk.

Our study has several strengths worth noting. In this first study to examine Cd body burden and GDM risk, we used a large and well-characterized cohort of pregnant women to complete our research. The prospective nature of the parent Omega Study facilitated the exclusion of women with diagnosed pregestational diabetes and renal disease, and the use of early-pregnancy biological samples allowed us to characterize Cd body burden during the critical period of early pregnancy when pathophysiologic changes of GDM are believed to start (Blackburn 2013). Urinary metals were assessed by a robust, well-validated, and accurate method (ICP-MS). Structured interviews, medical record abstraction, and a semiquantitative FFQ provided rich covariate data. In sum, our study and its findings provide new information to address a knowledge gap in the literature.

Our study is not without limitations and should be interpreted with caution due to the observed attenuation of effect between the primary analyses and the sensitivity analyses that included women with dilute urine. The WHO creatinine guidelines may be overly restrictive for women, because women tend to have lower creatinine levels than the male occupational cohorts upon which the guidelines were originally based (Barr et al. 2005). However, we are not aware of any published criteria specific to the assessment of creatinine in spot urine samples during pregnancy. Some prior research suggests that creatinine may be an independent predictor of diabetes mellitus (Yassine et al. 2012). However, in our analytic population, creatinine levels measured in early pregnancy were not different among women with and without GDM [geometric mean (GM) = 82.6 mg/dL; 95% CI: 75.3, 90.7 for GDM cases; GM = 83.6 mg/dL; 95% CI: 79.5, 87.9 for noncases]. Additionally, humans are exposed to complex mixtures of toxic substances every day, and as with all studies of environmental exposures, there is an inherent difficulty in singling out the effect of Cd. Therefore, unknown and unmeasured co-exposures may influence the risk of GDM. Because of the small sample size, we had limited statistical power for assessing potential effect modification. Although we did not observe effect modification by smoking status, we were unable to assess the effect of environmental tobacco smoke on the Cd-GDM relation. Generalizability of our findings may be somewhat reduced because women in the Omega study are generally non-Hispanic white, married, and affluent, reflective of the underlying population that uses Swedish Medical Center and Tacoma General Hospital. Our study population also represents a subgroup of the general population with average urinary creatinine-corrected Cd greater than among women in the general U.S. population as estimated by the NHANES (GM = 0.25 μg/g Cr; 95% CI: 0.24, 0.27) (Centers for Disease Control and Prevention 2013).

## Conclusions

Collectively, our findings suggest that Cd may be an important environmental risk factor for GDM. Replication of these findings in other studies, especially studies with more ethnically diverse populations, will be important to gain a fuller understanding of the association between Cd body burden and GDM. Ultimately, improved understanding of GDM-related environmental risk factors, particularly those that are modifiable, will assist in identifying women at higher risk of GDM and provide preventative opportunities.
